The article "A Study on Fucosyltransferase 2 Gene Polymorphism and Secretion Status Related to Neonatal Necrotizing Enterocolitis" was retracted in 2023. Reasons: signs of a paper mill; suspected computer-generated content; unreliable results or conclusions; concerns about the data.

# A Study on Fucosyltransferase 2 Gene Polymorphism and Secretion Status Related to Neonatal Necrotizing Enterocolitis

**DOI:** 10.1155/2021/7219850

**Published:** 2021-07-21

**Authors:** Qing Ye, Jialin Yu

**Affiliations:** ^1^Department of Neonatology, Children's Hospital of Chongqing Medical University, Chongqing 400014, China; ^2^Department of Pediatrics, Shenzhen University General Hospital, Shenzhen 518055, Guangdong, China

## Abstract

**Objective:**

To detect the single nucleotide polymorphism (SNP) of alpha-(1,2) fucosyltransferase 2 gene (FUT2) and the secretion status in the newborns of Chongqing China and explore the relationship between genotype or phenotype of FUT2 and neonatal necrotizing enterocolitis (NEC).

**Methods:**

Newborns who were hospitalized in Children's Hospital of Chongqing Medical University from August 2014 to December 2015 and in line with the inclusion criteria were chosen as the research subjects; 34 cases of them in accordance with the diagnostic criteria of NEC stage II or III were NEC group, and 36 other cases of them were the control group. Total DNA was extracted from oral epithelial cells of patients which were collected with cotton buds. FUT2 SNP genotype was detected by gene sequencing. H antigen was detected with saliva samples by saliva agglutination inhibition test. Related clinical data were collected for analysis.

**Results:**

There are three genotypes on the rs1047781 (A385T) allele of the FUT2 encoding sequence: AA, AT, and TT. The number of genotypes AA, AT, and TT in the NEC group was 9 (26.47%), 12 (35.29%), and 13 (38.24%), respectively. In the control group, the number of genotypes AA, AT, and TT was 12 (33.33%), 17 (47.23%), and 7 (19.44%). There were no differences in genotypes between the two groups according to the chi-square test (*P* > 0.05). There were 22 cases of secretors (64.7%) and 12 cases of nonsecretors (35.3%) in the NEC group. The number of secretors and nonsecretors in the control group was 31 (88.89%) and 5 (11.11%). Statistical difference was found in the phenotype between two groups through the chi-square test (*P* < 0.05). In addition, no G428A homozygous mutation, which causes nonsecretor phenotype in Caucasians, was seen in all the subjects of this study.

**Conclusions:**

These findings indicate that secretion status (nonsecretor) was significantly associated with NEC in Chongqing, China.

## 1. Introduction

Neonatal necrotizing enterocolitis (NEC) is an acute abdomen disorder in the neonatal period. It is more common in premature infants, with a fatality rate as high as 50% [1, 2]. Most of the surviving children have serious sequelae. It threatens the survival and health of newborns. Since the exact cause of the disease is still unclear, it is very urgent to clarify the pathogenesis of NEC to prevent the disease. At present, NEC is considered as a multifactorial disease, closely related to gestational age, birth weight, birth mode, feeding mode, and changes in the gut microbiota of neonates. Studies show that the occurrence of NEC in neonates is related to changes in gut microbiota [3, 4]. Plummer et al. also reported that increased abundance of *Bifidobacterium* soon after birth may be associated with reducing the risk of NEC in very preterm infants [5]. The polysaccharides in the intestinal epithelium and their secretions in the intestinal mucosa are the ones that have the closest contact with the gut microbiota [6, 7].

Histoblood group antigens (HBGAs) are ABH blood group antigens found in body fluids and some epithelial tissues. They are a series of polyglycoprotein substances formed after fucosylation mediated by *α*-(1,2) fucosyltransferase encoded by the FUT2 gene. She et al. have examined paraffin-embedded intestinal specimens from participants and found that the NEC patients showed lower intestinal epithelial fucosylation levels than the control patients [8]. At the same time, studies have shown that fucosylation of intestinal epithelial cells participates in the maintenance of gut microbiota homeostasis, and it is also of great significance in the colonization of intestinal symbiotic bacteria [9, 10].

These studies provide us with new ideas for exploring the pathogenesis and prevention of NEC. Are fucosylation and histoblood group antigen, which are closely related to gut microbiota, related to NEC? At the same time, the target population of the above studies is all Caucasian, and the key site of the FUT2 gene, which determines secretor phenotype, is different in different races. So far, there has not been any research that shows that FUT2 genotypes or phenotypes are associated with NEC in the Chinese population. Therefore, this study is intended to understand the SNP sites which control the secretion status of the FUT2 in the population of Chongqing in China and to explore the relationship between FUT2 genotype or phenotype and neonatal necrotizing enterocolitis (NEC) by detecting the genotypes and phenotypes of FUT2 of newborns.

## 2. Research Subjects and Methods

### 2.1. Materials

#### 2.1.1. Research Subjects

1. Specimen source: specimens were collected from the newborns who were hospitalized in Children's Hospital of Chongqing Medical University from August 2014 to December 2015.
2. To be included in the NEC group, the specimen must meet the following two requirements at the same time: ① NEC diagnosis should meet the revised Bell's NEC II or III clinical diagnostic criteria [11]; ② newborns with gastrointestinal malformations and inflammation should be excluded.
3. The control group should meet the following conditions at the same time: ① non-NEC newborns were admitted to our hospital at the same time; ② newborns with gastrointestinal malformation, inflammation, sepsis, severe anemia, disseminated intravascular coagulation (DIC), and congenital malformation of the respiratory tract, heart, brain, and kidney were excluded; ③ gestational age, birth weight, and feeding pattern were matched with the NEC group.
4. Subgroup grouping: ① NEC cases were divided into AA, AT, and TT subgroups according to the sequencing results of FUT2 SNP rs1047781. ② NEC cases were divided into secretor and nonsecretor subgroups according to the detection of histoblood group antigens in saliva.
5. The treatment principles of the two groups were as follows: the NEC group needed to fast after admission. The newborns in the control group and those NEC patients after the resumption of feeding were fed with the same formula milk.
6. Sample collecting: ① according to previous studies, the histoblood group antigens in the saliva of newborns gradually increased in the first week after birth, and the endocrine level was basically flat in the second week after birth. Therefore, in this study, saliva samples were collected from newborns with the NEC group and control group over 7 days of age. ② Saliva samples were collected between 19 to 22 o'clock and at least 1 hour after eating. ③ Samples were collected in a unified way.
7. This study was approved by the Ethics Committee of Children's Hospital of Chongqing Medical University, and the family members were informed and signed the consent form.

#### 2.1.2. Preparation and Storage of Samples

1. Oral epithelial cells of patients were collected with sterile cotton buds and stored frozen at −80°C until tested.
2. Sterile cotton swab was placed in newborn's mouth, saturated with saliva, removed and placed in a 1.5 mL centrifuge tube, 0.5 mL of normal saline added and centrifuged at 1000*g* with 10 minutes. Then, the supernatant was collected and boiled in water for 10 minutes to inactivate saliva enzymes. After centrifuging at 10 minutes, the clear or slightly milky white supernatant was collected as the prepared saliva and discarded the opaque or semisolid substances. If the prepared saliva is used within a few hours, it can be stored at 4°C; if it is used after more than 1 day, it must be stored frozen at −20°C (the activity can remain constant for several years).

### 2.2. Methods

#### 2.2.1. DNA Extraction of Oral Swab Epithelial Cells

DNA extraction procedures of oral swab epithelial cells were followed by the instructions for QIAAMP DNA Investigator56504 (QIAGEN, Germany). The DNA was divided into 3 tubes (30 *μ*l, 30 *μ*l, and 30 *μ*l, respectively) and stored in a refrigerator at −80°C.

#### 2.2.2. PCR Amplification and Product Detection

(1) PCR amplification: PCR amplification was performed with forward and reverse primers of FUT2 gene (Shanghai Sangon)—forward F (5′-AGCGCCCCGGGCCTCCATCTCC-3′) and reverse R (5′-GGAACCATGTGCTTCTCATGCCCG-3′). The reaction system and conditions are as follows.

#### 2.2.3. SNP Site Detection of FUT2 Gene

1. 20 *μ*l of the PCR product was packed in an icebox and sent to Shanghai Bioengineering Department for sequencing
2. The corresponding SNP site polymorphisms (Table 1) were analyzed according to the sequencing map

#### 2.2.4. Detection of ABH Antigens in Saliva

1. Twelve small test tubes were taken and divided into groups A, B, and H, with 4 tubes in each group, which were marked respectively as a negative control, positive control, saline control, and tested tube.
2. At first, 20 *μ*l of anti-A, B, and H reagents corresponding to this group were added into each tube of the three labeled groups. Then, 20 *μ*l of normal saline was added to the saline control tube; 20 *μ*l of nonsecretory saliva to the negative control tube; 20 *μ*l of secretory saliva to the positive control tube; 20 *μ*l of the subject's saliva to the tested tube.
3. Incubate at room temperature for 30 to 60 minutes, shaking several times during the period to neutralize fully.
4. Each tube was added with 20 *μ*l of the corresponding 2%–5% reagent red blood cell (indicator red blood cell) suspension. Type A red blood cells were added to group A, type B red blood cells to group B, and type O red blood cells to group H.
5. Mix well, centrifuge immediately at 1000*g* for 1 min, and transfer to a microscope to observe the results.
6. Judgment of the results: agglutination occurred in negative control and saline pair, while no agglutination occurred in positive pair, indicating normal test.

Agglutination occurred in negative control and saline pairs, but not in positive pairs, and the test tube has agglutination, indicating that the antibody in the reagent serum has not been inhibited or neutralized, and it can still react with the indicator red blood cells. So, the saliva tested does not contain the corresponding blood group substances, and it is judged as a nonsecreted type.

Agglutination appeared in negative control and saline pair, but not in the positive pair, nor in the tested tube, indicating that the antibody in reagent serum was neutralized or inhibited and could not react with indicator red blood cells. This may demonstrate that there are corresponding blood group substances in the saliva and that it can be determined as the secretory type.

### 2.3. SNP Site Analysis of FUT2 Gene

The chromas software was used to read the sequencing peak map, and three SNP loci (rs1047781, rs281377, and rs601338) on the FUT2 gene were selected for analysis.

### 2.4. Analysis of Secretion Types

The secretor is defined as those with at least one ABH blood antigens detected in their saliva, while the nonsecretor is defined as those with no ABH blood group antigens detected in their saliva.

### 2.5. Statistical Methods

All data were calculated by SPSS21.0 statistical software, and the measurement data conform to the normal distribution, expressed by mean and standard deviation; the comparison between groups is made by *t*-test; the measurement data do not conform to the normal distribution, the rank sum test is used; the count data is between groups. The chi-square test was used for comparison, and the test level *α* was 0.05. When *P* < 0.05, it was statistically significant.

## 3. Research Results

### 3.1. The General Situation

The study subjects involve 34 NEC newborns and 36 newborns in the control group who met the inclusion criteria, with a total of 70 samples. There was no statistical significance in gender composition, gestational age, and birth weight between the two groups (see Table 2 for details).

### 3.2. SNP Site Results of FUT2 Gene

In this study, a total of 34 cases of the NEC group and 36 cases of the control group were successfully sequenced and analyzed. The genotype distribution of FUT2 gene rs1047781 (A385T), rs281377 (C357T), and rs601338 (G428A) was in line with Hardy–Weinberg equilibrium. Among them, there were AA, AT, and TT genotypes at the A385T site. At the C357T site, only heterozygous mutant CT and homozygous mutant TT genotypes were detected in the samples in this study. G428A is a key site that determines the secretory state in Caucasians. No such mutation was detected in this study, and all genotypes were GG (Figures 1–6 show the sequence diagrams of each allele of the three sites).

Table 3 shows the detailed results of sequencing. Among them, there are three genotypes, AA, AT, and TT, AT A385T site, which is considered to be the key locus that determines the secretion type of the Asian population. The C357T site is a common meaningless mutation site in the Asian population. There are two genotypes, CT and TT, in this test. G428A is a key site that determines secretion type in Caucasians. No such mutation was detected in this study, and all samples were GG (see Table 3 for details).

### 3.3. Histoblood Group Antigen Secretion Type Results

#### 3.3.1. Cases of Neonatal Secretion Type

In the study, a total of 34 cases of the NEC group and 36 cases of the control group were successfully detected and analyzed. In the NEC group, 12 newborns (35.29%) were nonsecretors, while in the control group, 5 newborns (13.89%) were nonsecretors. The difference between the two groups was statistically significant (*χ*^2^ = 4.357, *P*=0.037). All the nonsecretor genotypes were TT homozygous mutation AT A385T site, and all the newborns with A allele (genotype AA and AT) in the experiment were secretors, which suggests that A385T is a key site controlling secretion type. However, though we found a total of 3 newborns (1 in the NEC group and 2 in the control group) whose genotype was TT homozygous mutation, yet histoblood group antigens were detected in their saliva, whereby it could be defined as the secretion type (see Table 4 for details).

#### 3.3.2. Comparison of Clinical Data

According to the secretion type, 34 people in the NEC group were divided into two subgroups: the secretors N1 group and the nonsecretors N2 group, and the corresponding clinical data were collected and analyzed. WBC, CRP, hsCRP, and PCT were the maximum values of each newborn examined during hospitalization, and the average or median values were calculated. Days of onset were defined as the number of days the child fasted (see Table 5 for details).

In the subgroups of the secretors and the nonsecretors groups, statistics about gender, gestational age, birth weight, white blood cells, CRP, allergic CRP and PCT, and the number of days being ill has shown that the indexes related to inflammation tends to be higher in the nonsecretors group than in the secretors group, especially the PCT of the nonsecretors group (median); it is 2.65 times as high as that of the secretors group. But this difference was not statistically significant.

## 4. Discussion

As a type of carbohydrate and a complex of some oligosaccharides and proteins or fatty acids, histoblood group antigens (HBGAs) are distributed on the surface of red blood cells, intestinal and respiratory epithelia and can also exist as free antigens in body fluids, such as in saliva, breast milk, and digestive juices. It is produced by adding fucose to the *α*-(1,2) position of its precursor to produce H antigen, which is catalyzed by *α*-(1,2) fucosyltransferase. In human beings, two kinds of *α*-(1,2) fucosyltransferases are known to be involved in the synthesis of these antigens. They are encoded by two different genes, FUT1 and FUT2 genes. The FUT1 gene mainly determines the antigens on red blood cells, while the FUT2 gene mainly determines the antigens of other mucosal tissues and epithelial cells. Individuals with FUT2 gene-positive under the action of FUT2 gene add fucose on the precursor through *α*-(1,2) fucosyltransferase to form H antigen. On this basis, A, B, and Lewis antigens are formed in their body fluids and various epithelial cells. Thus, they are called “secretors.” If there is a mutation in the gene site encoding the enzyme on FUT2, the homozygous mutant individuals cannot form H antigen and consequently cannot form A, B, and Lewis antigens in the body fluids and various epithelial cells. They are called “nonsecretors.”

According to some current reports [12], the SNP sites on the FUT2 gene, including Se357, Se385, Se428, Se480, and Se739, have been identified in different ethnic groups. Among them, rs601338 (G428A, Se428) mainly determines the Nonsecretors of Caucasians. This is because the mutations of G>A at site 428 lead to an early stop codon, so it is unable to produce a functional *α*-(1,2) fucosyltransferase, resulting in nonsecretors. In the Chongqing Han population of China, rs1047781 (A385T, Se385) is the most common single nucleotide polymorphism that causes individuals nonsecretor [13]. There are 3 genotypes of AA, AT, and TT at the A385T site. People with TT genotype as a result of homozygous mutations are theoretically regarded as nonsecretor individuals. But not all individuals with homozygous mutations in TT are nonsecretors. From the results of the study, all individuals with A alleles (AA and AT) are secretors. However, 3 infants (1 in the NEC group and 2 in the control group) with homozygous TT mutations also detected histoblood group antigens in their saliva and were judged to be secretors. This is because A385T is a missense mutation at position 385 (A > T) that changes amino acid 129 from isoleucine to phenylalanine. The enzyme encoded by the gene containing the mutation is unstable and more easily hydrolyzed, making the amount of this enzyme significantly less than that of the wild-type enzyme, resulting in a weakly secreted or nonsecreted state [14]. Homozygous carriers of this mutation led to nonsecretors or weak secretors, and ABH blood group substances cannot be detected in their saliva. This genetic mutation is widespread in Southeast and East Asian countries [15]. However, the degree of this hydrolysis may vary between individuals. In some populations, the hydrolysis is not complete, so the H antigen can also be detected in some homozygous mutant individuals [16].

Current studies have shown that the secretion status of histoblood group antigens is related to many infectious diseases. Secretors are more susceptible to norovirus [17, 18], *Helicobacter pylori* [19], influenza virus, rhinovirus, respiratory syncytial virus, and echovirus, but are less susceptible to haemophilus, meningitis dicoccus, *Streptococcus pneumoniae*, *Candida albicans* infection, and *E. coli*-induced urinary tract infections. The antigens can be used as a receptor for bacteria or viruses to bind and colonize, enabling them to have a certain connection with the fixed value of bacteria or related antibacterial effects [20, 21]. Histoblood group antigens gradually increase in the first week after birth [22], and the first week is also an important period for neonatal intestinal bacterial colonization. Some symbiotic bacteria (such as Bacteroides, etc.) can produce fucosidase, which separates and binds fucose groups from the surface of epithelial cells. The bound L-fucose is catabolized and metabolized by a series of fucose degrading enzymes, which can ① be used as energy for bacteria; ② be internalized into fucosylated capsular polysaccharides (components of the bacterial cell wall); ③ be used to regulate the expression of fucose operon genes; ④ be used as raw material for bacteria to produce short-chain fatty acids (SCFAs). In addition, epithelial cell fucosylation can provide colonization advantages for bacteria containing fucosidase such as Bacteroides, increase the number of beneficial intestinal flora, and promote colonization resistance against opportunistic pathogens [9, 10]. Some other studies have also pointed out that the composition of adult gut microbiota is related to the secretion status determined by the FUT2 gene [23], and histoblood group antigens may be a crucial genetic factor affecting the microecology of the intestinal flora [24]. There is no definite answer to the cause of NEC. The gut microbiota has many important physiological functions and plays an important role in the digestion and absorption of nutrients and immune regulation. Its abnormal colonization is one of the mechanisms leading to the occurrence of NEC [25]. Mshvildadze and Neu [26] also reported that NEC has lower bacterial diversity than the control group in the early stage of onset, and intestinal flora disorder is an important cause of its onset. In this study, there are more nonsecretors in the NEC group than in the control group (*P* < 0.05), so we guess that the nonsecretor or low-secreting newborns are susceptible to NEC, which is probably caused by affecting the intestinal flora.

FUT2 gene polymorphism is not only related to infectious diseases but also to the susceptibility of Crohn's disease [27, 28], primary sclerosing cholangitis [29], type 1 diabetes [30], and other autoimmune diseases. It is pointed out in the literature that the nonsecreting population is related to the susceptibility of Crohn's disease, which belongs to the same intestinal disease. At the same time, this may be caused by the changes of gut microbiota associated with histoblood group antigens. In this study, although 13 (38.24%) of the TT genes in the NEC group were more than 7 (19.44%) in the control group at the A385T locus, the difference was not statistically significant, yet this result may be caused by the insufficient sample size. The results need to be repeated and confirmed by a larger sample.

This study shows that the A385T gene polymorphism of the FUT2 gene may not be related to neonatal necrotizing enterocolitis in Chongqing, China. The nonsecretor is associated with neonatal necrotizing enterocolitis in Chongqing, China. This correlation may be caused by the secretion state affecting the gut microbiota of newborns. Admittedly, there still exist some shortcomings in this study. It is a single-centered and small-sample study, the number of included research subjects is limited, and the results obtained may be somewhat deviated from the real fact.

There is a longstanding interest in identifying contributors to and biomarkers of NEC in newborns. This study draws attention to the role of glycosylation. Related follow-up experiments on the microecological part will continue to be carried out to further explore the causes of NEC and to provide a reference for clinical prevention of NEC.

## Figures and Tables

**Figure 1:** Genotype TT on SNP rs1047781 (A385T).

**Figure 2:** Genotype AT on SNP rs1047781 (A385T).

**Figure 3:** Genotype AA on SNP rs1047781 (A385T).

**Figure 4:** Genotype TT on SNP rs281377 (C357T).

**Figure 5:** Genotype CT on SNP rs281377 (C357T).

**Figure 6:** Genotype GG on SNP rs601338 (G428A).

**Table 1:** Reaction system and conditions.

Reaction system	(50 *μ*l)	Conditions		
Template DNA	5 *μ*l	96°C	5 min	
Forward primer	1 *μ*l	95°C	20 s	13 cycles
Reverse primer	1 *μ*l	78°C	40 s	
Premix Taq	25 *μ*l	95°C	10 s	
ddH_2_O	18 *μ*l	62°C	10 s	25 cycles
Total	50 *μ*l	72°C	2 min	
		72°C	5 min	
		4°C	Termination reaction	

**Table 2:** Clinical data of NEC group and control group.

Grouping clinical features	NEC group	Control group	Statistics	*P* value
	*n* = 34	*n* = 36		
Gender (male/female)	(18/16)	(16/20)	*χ* ^2^ = 0.505	*P*=0.319
Gestational age ($\bar{x}\pm s,d$)	36.58 ± 3.22	37.20 ± 3.20	*t* = −0.81	*P*=0.42
Birth weight ($\bar{x}\pm s,d$)	2594.85 ± 952.88	2762.03 ± 836.66	*t* = −0.78	*P*=0.44

**Table 3:** Genotype of NEC and control group on allele A385T, C357T, G428A of FUT2.

SNP	Genotype	NEC group *n* (%)	Control group *n* (%)	Statistics	*P* value
A385T	AA	9 (26.47)	12 (33.33)	*χ* ^2^ = 4.154	*P*=0.125^●^
	AT	12 (35.29)	17 (47.22)		
	TT	13 (38.24)	7 (19.44)		
	AA + AT	21 (61.76)	29 (80.56)	*χ* ^2^ = 3.025	*P*=0.082^Δ^
	A allele	30 (44.12)	42 (58.33)	*χ* ^2^ = 2.829	*P*=0.065^☆^
	T allele	38 (55.88)	30 (41.67)		

C357T	CC	0 (0)	0 (0)		
	CT	7 (20.59)	4 (10.26)		
	TT	27 (79.41)	32 (89.74)	*χ* ^2^ = 1.186	*P*=0.276
	C allele	7 (10.29)	4 (5.56)		
	T allele	61 (89.71)	68 (94.44)	*χ* ^2^ = 1.085	*P*=0.234
G428A	GG	68 (100)	72 (100)		

Note. ^●^ comparing the three genotypes of the A385T locus in the NEC group and the control group, there is a certain difference in the genetic polymorphism composition of the two groups, but *P* > 0.05, with no statistical significance; ^Δ^ comparing the number of TT genotypes at the locus of A385T of the two groups, it was found that the NEC group had more homozygous mutant TT types than the control group, but *P* > 0.05, which was not statistically significant; ^☆^ comparing the number of A allele and T allele at the A385T locus of the two groups, *P* > 0.05, which was not statistically significant.

**Table 4:** Secretor status of NEC and control group.

Group genotype	Secretors			Nonsecretors		
	AA + AT	TT	Total	AA + AT	TT	Total
NEC group	21	1	22 (64.71)	0	12	12 (35.29)
Control group	29	2	31 (86.11)	0	5	5 (13.89)
Statistics	*χ*2		4.357			
*P* value	*P*		0.037^▼^			

Note. ^▼^ comparing the number of secretors and nonsecretors of the two groups, it was found that the NEC group had more nonsecretors than the control group (*P* < 0.05).

**Table 5:** Clinical data of secretor group and nonsecretor group.

Grouping (total 34 cases)	Secretors	Nonsecretors	Statistics	*P* value
Clinical features	*N*1 = 22	*N*2 = 12		
Gender (male/female)	(9/13)	(9/3)	*χ* ^2^ = 3.62	*P*=0.08
Gestational age ($\bar{x}\pm s,d$)	36.46 ± 3.16	36.78 ± 3.46	*t* = −0.27	*P*=0.79
Birth weight ($\bar{x}\pm s,d$)	2515.00 ± 1079.89	2741.25 ± 679.34	*t* = −0.66	*P*=0.52
WBC ($\bar{x}\pm s,d$)	17.24 ± 8.15	18.27 ± 7.44	*t* = −0.37	*P*=0.71
CRP ($\bar{x}\pm s,d$)	40.16 ± 38.72	46.50 ± 36.69	*t* = −0.47	*P*=0.64
hsCRP ($\bar{x}\pm s,d$)	48.07 ± 49.75	67.30 ± 40.36	*t* = −1.06	*P*=0.296
The median of PCT (interquartile range (ng/ml))	1.20 (0.13∼3.37)	3.18 (0.54∼13.34)	*u* = 1.935	*P*=0.164
Days of onset ($\bar{x}\pm s,d$)	10.45 ± 5.27	11.09 ± 5.02	*t* = −0.34	*P*=0.74

## Data Availability

The data used to support the findings of this study are available from the corresponding author upon request.

## References

[1] Gerald W. (1990). Plasmid profiling of members of the family Enterobacteriaceae, lactobacilli and bifidobacteria to study the transmission of bacteria from mother to infants. *American Society Microbiology*.

[2] Torun M. M., Bahar H., Gür E., Taştan Y., Alikaşifoğlu M., Arvas A. (2002). Anaerobic fecal flora in healthy breast-fed Turkish babies born by different methods. *Anaerobe*.

[3] Elgin T. G., Kern S. L., Mcelroy S. J. (2016). Development of the neonatal intestinal microbiome and its association with necrotizing enterocolitis. *Clinical Therapeutics*.

[4] Xiao G. Z., Li J., Yi W.-h., Luo J.-j., Su L. (2017). Influence of glutamine on barrier function of heat-stressed intestinal epithelial caco-2 cells. *Medical Journal of Chinese People’s Liberation Army*.

[5] Plummer E. L., Bulach D. M., Murray G. L. (2018). Gut microbiota of preterm infants supplemented with probiotics: sub-study of the ProPrems trial. *BMC Microbiology*.

[6] Li Z. G., Jiang H. Y., Li L. J. (2015). Expression of Gal-9 in peripheral blood and colonic epithelial tissue of mice with colitis. *Journal of Zhengzhou University*.

[7] Goto Y., Uematsu S., Kiyono H. (2016). Epithelial glycosylation in gut homeostasis and inflammation. *Nature Immunology*.

[8] She X., Du H., Yi C., He Y., Ai Q., Yu J. (2021). The decrease of fucosylation in intestinal epithelium is related to the development of necrotizing enterocolitis. *Molecular Immunology*.

[9] Pham T. A. N., Clare S., Goulding D. (2014). Epithelial IL-22RA1-mediated fucosylation promotes intestinal colonization resistance to an opportunistic pathogen. *Cell Host & Microbe*.

[10] Giampaoli O., Conta G., Calvani R., Miccheli A. (2020). Can the FUT2 nonsecretor phenotype associated with gut microbiota increase the children susceptibility for type 1 diabetes? A mini review. *Frontiers in Nutrition*.

[11] Gordon P. V., Swanson J. R., Attridge J. T., Clark R. (2007). Emerging trends in acquired neonatal intestinal disease: is it time to abandon Bell’s criteria?. *Journal of Perinatology*.

[12] Kelly R. J., Rouquier S., Giorgi D., Lennon G. G., Lowe J. B. (1995). Sequence and expression of a candidate for the human secretor blood group *α* (1,2) fucosyltransferase gene (FUT2). *Journal of Biological Chemistry*.

[13] Liu Y.-H., Koda Y., Soejima M. (1999). The fusion gene at the ABO-secretor locus (FUT2): absence in Chinese populations. *Journal of Human Genetics*.

[14] Chang J. G., Ko Y. C., Lee J. C. (2008). Molecular analysis of mutations and polymorphisms of the Lewis secretor type alpha (1,2)-fucosyltransferase gene reveals that Taiwan aborigines are of Austronesian derivation. *J Human Genetics*.

[15] Ferrer-Admetlla A., Sikora M., Laayouni H. (2009). A natural history of FUT2 polymorphism in humans. *Molecular Biology and Evolution*.

[16] Henry S. (2014). The Se(w) FUT2 mutation A385T does not result in a non-secretor allele. *Transfusion*.

[17] Currier R. L., Payne D. C., Staat M. A. (2015). Innate susceptibility to norovirus infections influenced by FUT2 genotype in a United States pediatric population. *Clinical Infectious Diseases*.

[18] Liu P., Wang X., Lee J.-C. (2014). Genetic susceptibility to norovirus GII.3 and GII.4 infections in Chinese pediatric diarrheal disease. *Pediatric Infectious Disease Journal*.

[19] Lindén S., Mahdavi J., Semino-Mora C. (2008). Role of ABO secretor status in mucosal innate immunity and H. pylori infection. *PLoS Pathogens*.

[20] Meng D., Newburg D. S., Young C. (2007). Bacterial symbionts induce a FUT2-dependent fucosylated niche on colonic epithelium via ERK and JNK signaling. *American Journal of Physiology-Gastrointestinal and Liver Physiology*.

[21] Nanda Nanthakumar N., Dai D., Newburg D. S., Allan Walker W. (2003). The role of indigenous microflora in the development of murine intestinal fucosyl‐ and sialyltransferases. *The FASEB Journal*.

[22] Morrow A. L., Meinzen-Derr J., Huang P. (2011). Fucosyltransferase 2 nonsecretor and low secretor status predicts severe outcomes in premature infants. *The Journal of Pediatrics*.

[23] Wacklin P., Tuimala J., Nikkilä J. (2014). Faecal microbiota composition in adults is associated with the FUT2 gene determining the secretor status. *PLoS One*.

[24] Wacklin P., Mäkivuokko H., Alakulppi N. (2011). Secretor genotype (FUT2 gene) is strongly associated with the composition of Bifidobacteria in the human intestine. *PLoS One*.

[25] Patel R. M., Denning P. W. (2015). Intestinal microbiota and its relationship with necrotizing enterocolitis. *Pediatric Research*.

[26] Mshvildadze M., Neu J. (2009). Probiotics and prevention of necrotizing enterocolitis. *Early Human Development*.

[27] Rausch P., Rehman A., Künzel S. (2011). Colonic mucosa-associated microbiota is influenced by an interaction of Crohn disease and FUT2 (secretor) genotype. *Proceedings of the National Academy of Sciences of the United States of America*.

[28] MeGovern D. P., Jones M. R., Taylor K. D. (2010). Fucosyltransferase2 (FUT2) non- secretor status is associated with Crohn’s disease. *Human Molecular Genetics*.

[29] Rupp C., Friedrich K., Folseraas T. (2014). Fut2genotype is a risk factor for dominant stenosis and biliary candida infections in primary sclerosing cholangitis. *Alimentary Pharmacology & Therapeutics*.

[30] Smyth D. J., Cooper J. D., Howson J. M. M. (2011). FUT2 nonsecretor status links type 1 diabetes susceptibility and resistance to infection. *Diabetes*.

